The article "Emphysematous cystitis and emphysematous pyelitis: a clinically misleading association" was retracted in 2015. Reason: plagiarism.

# Emphysematous cystitis and emphysematous pyelitis: a clinically misleading association

**DOI:** 10.11604/pamj.2013.16.18.2505

**Published:** 2013-09-17

**Authors:** Mustapha Ahsaini, Amadou Kassogue, Mohammed Fadl Tazi, Anas Zaougui, Jalal Edine Elammari, Abdelhak Khallouk, Mohammed Jamal El Fassi, My Hassan Farih

**Affiliations:** 1 Department of Urology, University Hospital Center Hassan II – FES, Morocco

**Keywords:** Diabetic, urinary tract infection, Emphysematous cystitis, computed tomography, bladder catherization

## Abstract

We present a rare case of emphysematous cystitis associated with an emphysematous pyelonephritis in a diabetic Arab man who was admitted in a confusional state. A 60-year-old man was admitted to the emergency department with confusion and hypogastric mass. The Clinical examination found comatose patient with a mass in the tympanic hypogastric percussion. The pelvic computed tomography (CT) demonstrated intramural gas in the urinarytract, which suggested a diagnosis of emphysematous cystitis and emphysematous pyelitis. The treatment was based on an antibiotics associated with a bladder drainage and diabetes stabilization. The evolution was uneventful. Every diabetic patient with a urinary tract infection who seems to be severely ill should have an abdominal X-ray as a minimal screening tool to detect emphysematous complications. The rarity and the association with an emphysematous pyelitis, which is rarely reported in the literature, are two remarkable characteristics described in this case report.

## Introduction

Emphysematous cystitis (EC) is the presence of intramural gas, with or without luminal gas, within the bladder as a result of a primary infection of the lower urinary tract with a gas-producing organism. The spectrum of clinical presentation of EC is non-specific and can range from minimally symptomatic urinary tract infection to a scenario of peritonitis and septic shock [1]. We report the case of EC associated with emphysematous pyelitis (EP) in a patient with diabetic tympani on hypogastric dullness.

## Patient and observation

A 60-year-old man, known diabetic, was admitted in emergency for disorders of consciousness. The medical history with the family revealed a notion of diabetes for 1 year and transurethral resection of the prostate for 5 years. A disorder of micturition for one year with burning urination. The examination found a feverish patient (38°C), a tympanic globe bladder and a prostate estimated to be 30g.

The biological balance sheet revealed an infectious syndrome with renal insufficiency (creatininemia = 57 mg/dl, CRP = 322 mg/dl, urea = 2.22 g/dl and a hyperglycemia = 6g/dl). Abdominal X-ray without preparation shows the presence of air (sight) at the pelvic area (Figure 1). Ultra-sonography (US) of the bladder was realized but was not contributive. An abdominal pelvic computed tomography (CT) without injection of intravenous contrast showed a vesical globe containing air (Figure 2, Figure 3) and the presence of the sight at the level of the left pyelon (Figure 4) confirming the diagnosis of cystitis and pyelonephritis emphysematous.

The article "Emphysematous cystitis and emphysematous pyelitis: a clinically misleading association" was retracted in 2015. Reason: plagiarism.

**Figure 1:** Urinary tract X-ray without preparation: showing air in the bladder region

**Figure 2:** Pelvic computed tomography (CT) shows a hydroaeric level and a pneumo bladder with air bubbles at the level of the vesical wall

**Figure 3:** Computed tomography scan of the pelvic shows air bubbles at the level of the vesical wall

**Figure 4:** The computed tomography scan with the arrow pointing to the emphysematous pyelitis

After a failure of urethral catheterization, the patient underwent a pubic catheterization returning gases and shady urines, drainage of the upper urinary tract was not done because of the lack of the expansion. Antibiotic treatment with ceftriaxone associated to metronidazole was started with an adapted insulotherapy. The bacterial culture of urines isolated an infection due to *Escherichia coli*. Apyrexy was obtained in 48 hours and a normalization of the renal function in 4 days. Urethrocystography retrograde micturition was realized after 3 weeks showing a stenosis of the urethra and the patient underwent an endoscopic uretrotomy.

## Discussion

Emphysematous cystitis is a rare disease mostly in the patients in their late fifties. It is twice as frequent in women as in men [2]. It occurs mainly in the elderly with poorly controlled diabetes. Other predisposing factors include the presence of a post-micturition residue or chronic retention (neurogenic bladder, diabetic, prostatic or urethral obstacle), presence of renal transplantation, renal infarction, systemic lupus, immunodepression due to long-term corticotherapy or immunosuppressors such as cyclophosphamides well-known for their vesical toxicity, the occurrence of postoperative emphysematous cystitis following endoscopic urologic procedures or colic surgery have been reported in the literature [2].

The culprits are strict anaerobic germs such as *Clostridium perfringens*, which rarely affect the urinary tract, and therefore, are rarely incriminated in EC. EC often occurs after an infection by aerobic anaerobic optimal germs (*Escherichia Coli*, *Enterobacter ariginosa*, *Klebsiella pneumoniae*, *Proteus mirabilis*, *Staphylococus aureus*, Streptococci) [3, 2]. *Escherichia coli* is often involved in the emphysematous cystitis. This germ was isolated in 60% to 70% of the cases. The anaerobic germ is not found in haemocultures, because bacteriological research does not include a systematic use of anaerobic culture. Carbon dioxide (CO2) is the gas found in the vesical light and/or the wall. It results from the bacterial glucid fermentation and testifies to bacterial breathing in anaerobiosis. CO2 producing germs attack not only the glucose that is present in the urine of the diabetics, which causes air to appear in the bladder cavity, but also the glucose contained in the bladder parietal cells, which causes CO2 bubbles to appear inside the vesical wall [3].

The article "Emphysematous cystitis and emphysematous pyelitis: a clinically misleading association" was retracted in 2015. Reason: plagiarism.

Emphysematous cystitis associated with more extended urologic attacks together with the emphysematous ureteritis and emphysematous pyelonephritis or emphysematous prostates have been reported [2].

In our case, the EC was associated with an EP with a tympany to percussion hypogastric mass. Saw the failure of survey, cystostomy should be realized on a hypogastric mass tympany. We first realized a pelvic ultrasound that was inconclusive. An urinary tract X-ray without preparation which showed the presence of pelvic gas. We have completed on abdominopelvic CT scan without injection of intravenous contrast confirms the EC associated with EP. The presence of a hypogastric mass in a patient with tympany is confused as misleading.

The diagnosis of EC is confirmed more often by radiography. Therefore, radiography remains a cornerstone of positive and specific diagnosis of emphysematous cystitis. In view of the insights gained in a reclining patient, radiography without previous preparation of the abdomen shows a radio-transparent ring on the pelvis area, a pneumo bladder (edge clearly confirmed to the detrusor and dissecting the vesical wall) and a hydroaeric pelvic level [4]. The differential diagnosis is done with primitive pneumaturia defined by the presence of gas in the bladder and with or without passage into the urethra and, particularly, the communication of the bladder with hollow organs. The vesico-digestive fistulas (colic or grelic) can be diagnosed using the radiological digestive and vesical opacifications [2].

Treatment is based on three fundamental therapeutic principles: the first is drainage of the bladder using a transurethral probe or by supra pubic drain which removes the infected urine and gas, the upper urinay tract has not been drained because due to the lack of expansion; the second is taking samples and culturing the urine allows the institution of broad spectrum antibiotic treatment, which will be adapted by the data obtained. Initially the antibiotic therapy will be managed parenterally then replaced by oral medication to consolidate treatment. Finally, diabetes stabilization is necessary both for monitoring the condition and breaking the vicious circle the patient may find himself in. Hyperbasic oxygen treatment is not a standardized therapy attitude in this type of pathology, but it was associated with a clear clinical improvement [3].

The article "Emphysematous cystitis and emphysematous pyelitis: a clinically misleading association" was retracted in 2015. Reason: plagiarism.

The prognosis of EC and EP can be rather serious due to the therapeutic failures which can occur when there is an ignorance of the physiopathological mechanisms of EC and EP. Actually, the prognosis in the case of EC, EP remains good provided that it is diagnosed in time and that an effective treatment is started without any delay. In the event of serious sepsis, the disease can evolve into the complications of EC such as necrosis cystitis, emphysematous pyelonephritis, and despite antibiotic therapy, resuscitation and urine aspiration [5].

The EC and EP is a disease often occurring in the patients with poorly controlled diabetes. It most often results from an infection with either aerobe or anaerobe germs. The clinical picture remains non-specific in the majority of cases and amounts to a urinary infection. EC or EP diagnosis can be suspected by the clinical presence of a tympanic hypogastric mass, or septic state, and must be confirmed by radiology. The scanner is the examination of choice. Treatment of EC and EP is bladder drainage, or upper urinary tract drainage if there is an expansion, and an individualized antibiotic treatment plan.

## Conclusion

Emphysematous cystitis associated to emphysematous pyelonephritis is a severe form of urinary tract infection. The presence of a vesical globe with tympany should lead to the suspicion of emphysematous cystitis. The diagnosis and assessment of the extent of the lesion is confirmed by a CT scan. The gas and urine drainage must be quick to avoid vesical rupture and septic shock.
